The article "Component-Resolved Diagnostic Study of Egg Allergy in Northern Chinese Children" was retracted in 2024. Reasons: signs of a paper mill; suspected computer-generated content; unreliable results or conclusions; concerns about the data.

# Component-Resolved Diagnostic Study of Egg Allergy in Northern Chinese Children

**DOI:** 10.1155/2020/3831087

**Published:** 2020-03-11

**Authors:** Jiayi Zhang, Yongming Shen, Junpu Li, Huiqiang Li, Ping Si

**Affiliations:** ^1^Department of Medical Laboratory, Tianjin Children's Hospital, Tianjin, China; ^2^Department of Clinical Laboratory, Tianjin Chest Hospital, Tianjin, China; ^3^School of Medical Laboratory, Tianjin Medical University, Tianjin, China

## Abstract

**Background:**

Egg component-specific IgE can be useful to evaluate and diagnose egg allergy, but their prevalence and clinical significance remain unclear in the local population. Previous studies have led to contradictory results regarding the value of specific IgG and specific IgG4 in sensitization.

**Objective:**

We aimed to determine the level of specific IgE, IgG, and IgG4 antibodies to the major egg allergens in egg-allergic children.

**Methods:**

Children from 6 months to 10 years of age were recruited. Egg allergy was confirmed by either a strong clinical history or an increased egg white-sIgE level. Other allergies were diagnosed by reactivity to other allergens but without egg-related symptoms and history. The serum sIgE, sIgG, and sIgG4 levels to major egg allergenic components (Gal d 1, Gal d 2, Gal d 3, Gal d 4, and Gal d 5), sIgE level to egg white, and tIgE level were determined by light-initiated chemiluminescent assay (LICA), ELISA, or ImmunoCAP.

**Results:**

Egg-allergic children had significantly higher levels of sIgE, sIgG, and sIgG4 to egg components than nonallergic children. Gal d 2 was the predominant allergen, and Gal d 2 sIgE level correlated with the egg white-sIgE level. Ratios of sIgE/sIgG4 to egg components were highest before 1 year of age and dropped gradually in the first decade of life.

**Conclusion:**

Patterns of sIgE to egg components could distinguish different forms of egg allergy. Ratios of sIgE/sIgG4 could be useful in predicting tolerance in egg-sensitive subjects, but this needs further evaluation and investigation using more accurate models.

## 1. Introduction

Egg is one of the earliest food resources introduced during childhood, and egg allergy (EA) has become one of the most common pediatric food allergy problems globally. EA may include IgE- and/or non-IgE-mediated reactions, and it is estimated to affect 0.5-2% infants and children [1, 2]. The high prevalence is partly due to immature immune responses; hence, most EA children will develop clinical tolerance by school age. However, a small proportion of EA children's symptoms will persist and not be resolved until adolescence [3, 4].

The function of specific IgE (sIgE) in EA pathogenesis has been well described as the majority of symptoms of EA are related to IgE-related type I hypersensitivity reactions. As a widely used *in vitro* test, immunoassay of serum sIgE to egg has been proven to be an effective method to evaluate potential EA patients and to predict clinical reactions to oral food challenges with less exposure risks and less likelihood of interference from prior treatments [5].

Component-resolved diagnostics (CRD) have introduced the application of sIgE to allergen components and thus extended the allergen repertoire to a more precise sensitization profile [6]. Egg allergens are composed of more than 20 types of proteins and glycoproteins, among which the most predominant ones are Gal d 1 (ovomucoid), Gal d 2 (ovalbumin), Gal d 3 (ovotransferrin, conalbumin), Gal d 4 (egg white lysozyme) from egg white, and Gal d 5 (alpha-livetin) from egg yolk [7]. Gal d 1 is associated with allergy to heated egg and persistent allergy due to its stability in the presence of heat and proteinases, whereas other allergens, such as Gal d 2, are related to uncooked rather than cooked egg allergy [4]. Although the allergenicity of individual allergens has been investigated based on their molecular structures and biological properties, there is limited information about the diagnostic value of sIgE to egg components [8].

There are still ongoing debates concerning the function of specific IgG (sIgG) and specific IgG4 (sIgG4) during the process of EA, although sIgG is reported to trigger anaphylaxis as well [9]. Egg sIgG and sIgG4 are found in both atopic and healthy children, so they are not considered as recommended markers of allergic status [10, 11]. However, recent studies proposed that the sIgG4 or sIgE/sIgG4 ratio to egg or egg proteins could be a marker of tolerance either naturally occurring or after immunotherapy [12–14].

The aim of this study is to evaluate the polyisotypic responses to egg components for CRD in children from northern China and to investigate potential markers of sensitization and resolution in EA patients.

## 2. Materials and Methods

### 2.1. Subjects

130 children were included in this study, and all of whom were recruited from Tianjin Children's Hospital, China. The egg-allergic group included 56 children with typical symptoms (including cutaneous, respiratory, and gastrointestinal symptoms) and either a convincing history of clinical reaction after egg consumption (*n* = 13) or an increased egg-specific serum IgE level above 2 kU_A_/L (ImmunoCAP, Phadia, Uppsala, Sweden) (*n* = 43) [15]. The atopic group consisted of 39 patients with other allergen reactivities but no egg-related clinical symptoms and history, while the control subjects comprised 35 patients recruited from a surgical department with neither symptoms nor history of allergy. Due to the limited funding of our research and vulnerable relationship between clinicians and patients, provoking tests, like oral food challenges or skin prick test (SPT), were not conducted in our study. No subjects included in this study had received immunotherapy, such as glucocorticoid or antihistamine therapy. All recruited subjects who had received immunotherapy were excluded. There were no significant differences between groups in terms of age, gender, or ethnicity. Sera of all groups were collected at the time of study entry. The study was approved by the Ethics Committee of Tianjin Children's Hospital, and informed consent was obtained.

### 2.2. Determination of Total IgE and Egg-Specific IgE Levels

Total serum IgE and egg white-specific IgE levels were determined by using ImmunoCAP (Phadia, Uppsala, Sweden) and Phadia 250 system. Samples with sIgE to egg white ≥ 0.35 kU_A_/L were defined as positive.

### 2.3. Determination of Egg Component-Specific Immunoglobulin Levels

Specific IgE and specific IgG4 to egg components Gal d 1, Gal d 2, Gal d 3, Gal d 4, and Gal d 5 were determined by light-initiated chemiluminescent assay (LICA): methodological details are described elsewhere [16, 17]. The results of sIgE and sIgG4 were calculated as relative light units (RLU). The relative prevalence of single component-sIgE was calculated by comparing sIgE levels in the EA group with the mean value of sIgE levels in the atopic and control groups. The cutoff value was defined as two standard deviations above mean values for both the atopic and control groups.

Specific IgG to egg components Gal d 1, Gal d 2, Gal d 3, Gal d 4, and Gal d 5 were determined by ELISA. Gal d 1 (cat# T2011), Gal d 2 (cat# A5503), Gal d 3 (cat# C0755), and Gal d 4 (cat# L6876) were purchased from Sigma-Aldrich, USA. Gal d 5 (cat# CSA62) was purchased from Equitech-Bio, Inc., USA. Allergen-coated wells were prepared by adding 100 *μ*L phosphate-buffered saline- (PBS-) diluted (20 *μ*g/mL) allergen to each well of 96-well plates and incubating at 4°C overnight. Then, the plates were washed 3 times with PBS containing 0.05% Tween 20 (PBST), before blocking at 37°C for an hour with 150 *μ*L 3% bovine serum albumin (BSA). After that, 100 *μ*L PBST-diluted sera (1 : 20) were added to the plates and incubated for an hour at 37°C. Subsequently, plates were washed with PBST again, and 100 *μ*L horseradish peroxidase- (HRP-) conjugated anti-human IgG (purchased from Sigma-Aldrich, USA) (1 : 2000) diluted in PBST was added and incubated for 30 min at 37°C. 3,3′,5,5′-Tetramethylbenzidine (TMB) was added to develop the plates in the dark for 5 min, and 10% H_2_SO_4_ was added to terminate the reaction. OD values of the plates were measured at 450 nm immediately. The results of sIgG were calculated as the absorbance units (AU)/mL.

### 2.4. Statistical Analyses

Data and graphs were analyzed and generated by using GraphPad Prism 7 (GraphPad Software Inc., San Diego, CA, USA). Comparisons of general characteristics between groups were determined using Student's *t*-test, chi-square test (frequencies), and Kruskal-Wallis test.

Comparisons of sIgE, sIgG, and sIgG4 levels between groups were determined using the Kruskal-Wallis test. Once significant differences were found, the Mann-Whitney *U* test was performed to further evaluate differences between every two groups. Correlations were calculated with Spearman's rank order correlation coefficient test. A *p* value of *<*0.05 was considered to be statistically significant.

## 3. Results

### 3.1. Participants and Clinical History

Children in the egg-allergic, atopic, and control groups were similar in terms of age and gender. Members of the egg-allergic and other allergic groups had significantly higher total IgE levels and wider ranges of total IgE compared with control subjects. As expected, children in the egg-allergic group had a higher level of egg white-sIgE, whereas subjects in the other two groups had no detectable egg white-specific IgE (Table 1).

The most typical symptoms in egg allergy patients were cutaneous reactions, including eczema, urticaria, and other symptoms, which were observed in 30 (54%) children in this group.

Only a small proportion of patients presented with respiratory symptoms (asthma), gastrointestinal symptoms (diarrhea), and oral allergy syndromes (coughing and conjunctivitis) in the egg atopic group (Table 2). Of 56 egg-allergic children, 13 (23%) had reported a reaction to egg or egg-related food, and 7 (12%) had a parental history of atopy.

### 3.2. Egg Protein-Specific IgE Levels

Levels of sIgE to individual egg proteins were measured in all groups, whereas the allergenicity (IgE binding activity) was only determined in egg atopic participants. Patients with egg allergy had a significantly higher sIgE response to all 5 egg components than other atopic and nonatopic children, but these sIgE levels showed no statistical difference between other atopic and nonatopic patients (Figures 1(a)–1(e)). The higher sIgE relative values of EA children compared to other groups tended to be more significant in Gal d 2 and Gal d 3 than in other components (Figures 1(b) and 1(c)). Among the allergens in our study, Gal d 2 and Gal d 1 were the most allergenic, with 62.5% EA patients and 51.8% EA patients, respectively, showing a detectable sIgE. Of 56 EA children, 41.1% had detectable sIgE responses to Gal d 3, which were also higher compared with 14.3% to Gal d 4 and 23.2% to Gal d 5 (Figure 1(f)).

We found that in the EA group, Gal d 2 sIgE had the highest frequency of response in almost all egg component-sIgE screening-positive subjects (35 of 38, 92.1%). By contrast, Gal d 4 sIgE was only found in 3 patients with 4-type sIgE positive and 5 patients were allergic to all 5 components. And all participants who had Gal d 4 sIgE had a combination of sIgE to Gal d 1, Gal d 2, and Gal d 3. About one-third of the egg-allergic children (18 of 56, 32.1%) showed no IgE reaction to any of the 5 egg components examined (Table 3).

More than a half of the egg allergy patients (30 of 56, 53.6%) had more than one type of egg protein-specific IgE (Table 3), while only 8 children (14.3%) had one single detectable sIgE among the studied allergens (Figures 2(a) and 2(b)). Levels of egg white-sIgE correlated significantly with numbers of egg component-sIgE detected (*r* = 0.4876, *p* = 0.0001) and levels of Gal d 2 sIgE (*r* = 0.4855, *p* = 0.0001) in egg-atopic subjects (Figures 2(c) and 2(d)).

### 3.3. Egg Protein-Specific IgG and IgG4 Levels

Egg component protein-sIgG and sIgG4 levels were determined in all subjects. A significantly higher IgG response to allergens was seen among EA and atopic children versus nonatopic children. When compared with the atopic group, the EA group had a statistically higher sIgG level to all proteins except for Gal d 5 (Figure 3).

Children with EA had the highest levels of sIgG4 to Gal d 1 and Gal d 2 compared with the other two groups, and there is no statistical difference between other atopic and nonatopic subjects. For Gal d 3, Gal d 4, and Gal d 5, EA children had a higher sIgG4 response than nonatopic participants, whereas the difference between other atopic and egg-allergic subjects and between other atopic and nonatopic subjects was not significant (Figure 4).

### 3.4. Egg Protein-sIgE/sIgG4 Ratio among EA Children of Different Ages

In EA infants below 1 year old, sIgE/sIgG4 ratios to all egg components were similar in number (range: 3-9). After that, the sIgE/sIgG4 ratios of Gal d 1 and Gal d 2 dropped steeply in the early stage of childhood. Then, the trends began to decrease slowly until reaching a steady and low level (approximately 0.01) at around 6 years old. In contrast, the sIgE/sIgG4 ratios of components Gal d 3, Gal d 4, and Gal d 5 in EA children showed a slight drop before 4 years of age; then, the ratios remained steadily at about 0.3 for Gal d 3 and about 1 for Gal d 4 and Gal d 5. After 7 years old, Gal d 3, Gal d 4, and Gal d 5 sIgE/sIgG4 ratios began to decline to a lower level in EA patients (Figure 5).

## 4. Discussion

A bead-based light-initiated chemiluminescent assay (LICA) system was demonstrated in our previous studies to determine serum egg component-sIgE and sIgG4 profiles. LICA has been proven to have excellent analytical performances and a good correlation with Phadia ImmunoCAP tests in sIgE measurement [16, 17]. Yet, only a limited profile of allergy tests has been introduced in our country; LICA could be a reliable complement in allergy screening and diagnosis. The advent of component-resolved diagnostics (CRD) had eliminated the cross-reactivity of conventional allergen extract sIgE assays and brought more detailed perspectives in assessing sensitization [6]. By using LICA technology, specific immunoglobulin to allergenic egg proteins could be quantified to characterize immune responses in children with different sensitization statuses.

In our study, EA patients produced significantly more egg component-sIgE than other groups. The highest frequency of positive responses was seen in Gal d 1 and Gal d 2, while Gal d 4 sIgE was the least common in EA subjects. These results were comparable with other findings [18, 19]. A previous study has presented similar reactive rates to our results in egg-allergic patients [20], while another study showed more Gal d 1 sIgE cases than Gal d 2 [19]. This may be due to the different age ranges of the subjects, different cooking effects on egg allergenicity, timing of egg introduction, and racial differences. Another interesting finding of this study was that about a third of EA patients had no component-sIgE detected. The reasons for this might be that other egg components, not identified in our study, were involved, like ovomucin, prostaglandin D synthase, and cystatin from egg white or vitellenin (apovitellenin I) and apoprotein B (apovitellenin VI) from yolk [2]. Furthermore, this also indicates that although CRD can provide a more personalized sensitization pattern, it cannot yet substitute for allergen extracts-sIgE tests. Egg component-sIgG and sIgG4 were detected not only in EA subjects but also in the atopic group and the control group. This is consistent with findings from other studies [21]. Previous studies have proposed that levels of egg and Gal d 2 (ovalbumin) sIgG and sIgG4 had no significant difference in sensitive, tolerant, and control subjects [11, 22]. However, our results suggested that this might not necessarily be the case, as the EA group and the atopic group both had a higher component-sIgG level than nonatopic children. This is in line with the recent findings of IgE-sensitized children having more IgG responses due to induced gut permeability [10]. We further demonstrated that the EA group had higher egg protein-sIgG4 levels than the control group, which agreed with the work reported by Ruiter et al. [23]. Oral challenge tests were not performed in our study; thus, our EA patients might include allergic but tolerant individuals, and this could contribute to higher levels of sIgG4, which is regarded as an indicator of tolerance [12]. To identify the status of tolerance in egg-allergic children, egg protein-sIgE/sIgG4 ratios were investigated in previous studies [14, 24], and our study extended the findings to 5 egg proteins. The trends of sIgE/sIgG4 ratios were found to have association with the resolution process of egg allergy [4]. Also, the Gal d 2 (ovalbumin) sIgE/sIgG4 ratio, along with the skin prick test, has been reported to perform better in distinguishing both cooked and uncooked egg tolerance [14]. Therefore, further work is required to assess the clinical value of egg protein-sIgE/sIgG4 ratios in the local population.

In summary, egg protein component-sIgE can be predictive in egg allergy diagnostics and the allergenicity varies widely in each component. Although sIgG levels to egg proteins were not necessarily associated with egg sensitization, we proposed that component-sIgE/sIgG4 ratios could be promisingly indicative for monitoring the status of tolerance in EA patients. Furthermore, CRD can provide evidence for more accurate desensitization, more personalized dietary intervention and other patient-specific allergy management strategies. Future studies should be done to unveil key conformations of single allergens and to improve understanding about their allergenic mechanisms.

## Figures and Tables

**Figure 1:** sIgE levels to 5 types of egg protein components (Gal d 1-Gal d 5) in all groups (a–e) and prevalence of sIgE response in the EA group (f). Levels of specific IgE (RLU) to 5 types of egg allergy protein were measured in all subjects, and relative sIgE response was determined by comparing the data from the egg allergy group to the other two groups. *p* values were calculated with the Kruskal-Wallis test and Mann-Whitney *U* test, when appropriate. sIgE: specific IgE; NA: nonatopic; EA: egg allergy; A: atopic; NS: not significant; RLU: relative light units; ^∗^*p* < 0.01; ^∗∗^*p* < 0.001; ^∗∗∗^*p* < 0.0001; ^∗∗∗∗^*p* < 0.00001.

**Figure 2:** Prevalence of multicomponent-sIgE in children with egg allergy. The number of cases (a), proportion of cases (b), and egg white-sIgE (kU_A_/L) levels (c) with multiple types of protein-sIgE detected in the EA group. Correlation of Gal d 2 sIgE (RLU) levels (d) and egg white-sIgE (kU_A_/L) levels in EA patients. Correlations were calculated by using Spearman's rank order correlation coefficient test. sIgE: specific IgE; EA: egg allergy.

**Figure 3:** Egg protein components (Gal d 1-Gal d 5) sIgG levels in the A, EA, and NA groups (a–e) and comparison of antigenicity in all groups (f). Levels of specific IgG (AU/mL) to 5 types of egg allergy protein were determined and compared in all subjects. Boxes represent means and SDs of the values. *p* values were calculated by using the Kruskal-Wallis test and Mann-Whitney *U* test, when appropriate. sIgG: specific IgG; NA: nonatopic; EA: egg allergy; A: atopic; NS: not significant; ^∗^*p* < 0.01; ^∗∗^*p* < 0.001; ^∗∗∗^*p* < 0.0001; ^∗∗∗∗^*p* < 0.00001.

**Figure 4:** sIgG4 levels to 5 types of egg protein components (Gal d 1-Gal d 5) in all groups (a–e) and comparison of their relative values (f). Levels of specific IgG4 (RLU) to 5 types of egg components were determined and compared in all subjects. Boxes represent means and SDs of the values. *p* values were calculated using the Kruskal-Wallis test and Mann-Whitney *U* test, when appropriate. sIgG4: specific IgG4; NA: nonatopic; EA: egg allergy; A: atopic; RLU: relative light units; NS: not significant. ^∗^*p* < 0.01; ^∗∗^*p* < 0.001; ^∗∗∗^*p* < 0.0001; ^∗∗∗∗^*p* < 0.00001.

**Figure 5:** sIgE/sIgG4 ratios of single egg components in EA children (a–e) and comparison of means of sIgE/sIgG4 ratios in EA children (f) from 0 to 8 years of age. Ratios of reactions to 5 egg proteins were calculated by using paired data of sIgE and sIgG4 for each of the EA individuals and then plotted against their ages. Means and SD (not shown) of all 5 component ratios were determined in every age group and compared. Infants less than one year old were shown as age 0 in (f). sIgE: specific IgE; sIgG4: specific IgG4; EA: egg allergy; SD: standard deviation.

**Table 1:** Characteristics of other allergy, egg-allergy, and nonallergic subjects.

	Group A Other allergies	Group EA Egg allergy	Group NA Control	*p* value
*n*	39	56	35	
Age (y), median (range)	2.7 (0.5-8)	3.2 (0.5-8)	3 (0.5-10)	0.219
Male subjects, no. (%)	24 (61.5)	37 (66.1)	20 (57.1)	0.689
Total IgE (kU/L), median (range)	75 (2-1006)	193 (9-2166)	42 (2-312)	<0.001^∗∗^
Egg white-sIgE (kU_A_/L), median (range)	<0.35	1.4 (0.37-100)	<0.35	<0.001^∗∗^

*p* values were calculated by performing Student's *t*-test, chi-square test (frequencies), and Kruskal-Wallis test. The lower and upper limits of egg-sIgE detection assay are 0.35 and 100 kU_A_/L. A: atopic; EA: egg allergy; NA: nonatopic; sIgE: specific IgE.

**Table 2:** Summary of clinical manifestation of children in the egg-allergic group.

Symptoms	*N*	Frequency (%)
Eczema	14	25
Urticaria	10	17.9
Other skin symptoms	6	10.7
Asthma	3	5.4
Coughing	3	5.4
Diarrhea	3	5.4
Conjunctivitis	2	3.6

**Table 3:** Patterns of sensitization to egg components in children with EA (*N* = 56).

Types of sIgE detected	Pattern of sIgE combination	*N*
0	NA	18
1	Gal d 1	1
	Gal d 2	5
	Gal d 3	1
	Gal d 5	1
2	Gal d 1+Gal d 2	7
3	Gal d 1+Gal d 2+Gal d 3	8
	Gal d 1+Gal d 2+Gal d 5	1
	Gal d 2+Gal d 3+Gal d 5	2
4	Gal d 1+Gal d 2+Gal d 3+Gal d 4	3
	Gal d 1+Gal d 2+Gal d 3+Gal d 5	4
5	Gal d 1+Gal d 2+Gal d 3+Gal d 4+Gal d 5	5

## Data Availability

The data to support this study are available at the correspondence author upon request.

## Abbreviations

AU: Absorbance units
CRD: Component-resolved diagnostics
EA: Egg allergy
NA: Nonatopic
LICA: Light-initiated chemiluminescent assay
RLU: Relative light units
sIgE: Specific IgE
sIgG: Specific IgG
sIgG4: Specific IgG4
SPT: Skin prick test.
